# Risk Factors for Pulmonary Metastasis in Differentiated Thyroid Carcinoma Patients and the Significance of Changes in Matrix Metalloproteinase 13 and microRNA-142 Levels

**DOI:** 10.1155/2022/6820281

**Published:** 2022-09-05

**Authors:** Xiaoyang Zhang, Zhenqi Lu, Guannan Zhang, Shuai Li, Aiguo Zhao, Yayun Miao, Wensheng Wang

**Affiliations:** Breast and Thyroid Surgery Ward, The First Affiliated Hospital of Henan University, Kaifeng 475001, China

## Abstract

This work aims to explore the risk factors of lung metastasis (LM) in differentiated thyroid cancer (DTC) (LM-DTC) and the effect of treatment and to detect the relationship between LM-DTC and the levels of matrix metalloproteinase-13 (MMP-13) and micro ribonucleic acid (RNA)-142 (miR-142) in peripheral blood. The data of 420 patients with DTC who are admitted from March 2020 to December 2021 are collected and divided into a non-metastasis group (non-LM group) of 400 cases and metastasis group (LM group) of 20 cases according whether the mung metastasis is found. In addition, risk factors of LM-DTC are analysed and compared. The results of multivariate logistic analysis show that age, disease course, and imaging timing are independent influencing factors of the radionuclide treatment effect. Follicular carcinoma, abnormal expressions of MMP-13, and miR-142 can increase the risk of LM-DTC. MMP-13 and miR-142 can be undertaken as auxiliary diagnostic biological indicators.

## 1. Introduction

Thyroid cancer is a very common malignant tumor located in the endocrine system, and its incidence accounts for about 90% of endocrine malignant tumors and about 1% of systemic malignant tumors [1]. In recent years, the incidence of thyroid cancer in China has shown an upward trend year by year, ranking among the top 10 malignant tumors and the top 8 female malignant tumors, and the age of onset tends to be younger [2]. About 90% of thyroid cancers are differentiated thyroid cancer (DTC). DTC mainly originates from thyroid follicular epithelial cells, so most of them are papillary thyroid carcinoma and thyroid follicular cell carcinoma, and a few are eosinophilic tumors [3]. The disease progression of DTC is relatively slow and the prognosis of patients is good. Evidence shows that patients with DTC have a higher 10-year survival rate [4]. However, some DTCs progress rapidly, and distant metastasis occurs in cervical lymph nodes, lungs, and bone tissues. The rate of distant metastasis is 7% to 23%, but the 10-year survival rate of patients is only 40% [5]. The lung is the most common organ involved in DTC and the probability of lung metastasis (LM) in differentiated thyroid cancer (LM-DTC) ranges from 3% to 45% [6, 7]. The disease of LM-DTC is very insidious and has no specific clinical features, so it is the best time for treatment that has been delayed at the time of diagnosis. Therefore, early identification of DTC and LM is of great significance for improving the prognosis of patients [8, 9].

At present, the clinically recognized method for the treatment of DTC is mainly thyroid surgery combined with 131I radionuclide therapy combined with thyrotropin suppression therapy, and the recurrence rate after this method is reduced to 2.7%. Compared with surgical resection alone, the postoperative recurrence rate of combined treatment of DTC is reduced by about 30%. Studies have shown that with early diagnosis of DTC LM and aggressive treatment, the 10-year survival rate of patients can rise to 90%. However, the 2-year survival rate of patients who do not receive 131I radionuclide treatment is only 50%. 131I radionuclide treatment of DTC can uptake DTC lesions [10, 11]. The decay process of 131I can release beta rays, which can be directly used to kill tumor cells, thereby partially or completely eliminating the lesions and avoiding the recurrence or distant metastasis of DTC. 131I radionuclide in the treatment of DTC can significantly prolong the survival of patients and improve the quality of life of patients. However, the adverse reaction rate of 131I radionuclide in the treatment of DTC complicated with LM is high, such as acute emission lung injury.

The rest of this paper is organized as follows: Section 2 discusses related work.  Section 3 is the diagnostic criteria and treatment methods. The diagnostic efficacy and evaluation of clinical efficacy are discussed in Section 4.  Section 5 concludes the paper with summary.

## 2. Related Work

Thyroid cancer was a very common endocrine system malignant tumor, and its incidence accounted for more than 90% of endocrine tumors [12, 13]. First, the lesions of DTC patients with long disease courses were larger and the accumulation range expanded, which in turn led to distant metastasis of lungs and other tissues [14]. Follicular carcinoma was less differentiated than papillary carcinoma, and blood metastases were more common, making it more likely to develop LM. Cervical lymph node melanomametastasis (LNM) was also closely related to LM [15]. Other studies have confirmed that the probability of LM with positive mediastinal LNM was 5 times that of patients with negative LM [16]. Thyroid capsule invasion, endotracheal intubation (ETI), and mediastinal LNM all suggested that DTC was highly invasive and therefore more prone to distant metastasis [17].

The mechanism of tumor metastasis was very complex. When thyroid tumor cells metastasized, the extracellular matrix and basement membrane structure needed to be degraded first, and after breaking through the basement membrane structure, they transferred to other parts and form metastatic foci. Therefore, the process of tumor metastasis was regulated by various factors such as gene susceptibility and host affinity [18]. A variety of signalling pathways and cytokines were involved in the regulation of tumor cell metastasis. Matrix metalloproteinase-13 (MMP-13) was a member of the matrix metalloproteinase family, which could degrade the extracellular matrix and vascular basement membrane, so it played an important role in the local invasion and distant metastasis of tumor cells [19]. miR-142 was involved in various tumor processes, such as breast cancer, colorectal cancer and thyroid cancer, and its expression was downregulated [20, 21]. The results of this work showed that the expression level of MMP-13 in the serum of DTC LM patients was significantly upregulated, while the expression level of miR-142 was significantly decreased, suggesting that the expression of MMP-13 and miR-142 might be related to LM-DTC. Wang et al. confirmed that the expression of MMP-13 was upregulated in thyroid cancer with regional lymph node metastasis and was associated with TNM staging and recurrence of thyroid cancer [22]. Zhang et al. confirmed that miR-142-5p was involved in the regulation of epithelial-mesenchymal transition in the process of lung cancer cell metastasis and inhibits the metastasis of lung cancer [23]. Patients with longer disease courses had more distant metastases involving more organs and more metastases [24]. In the process of 131I treatment, 2% to 5% of DTC LM patients would have the performance of weakened iodine uptake and enhanced ability of distant metastasis. Therefore, the imaging timing of LM also affected the effect of 131I treatment of DTC LM [25, 26].

## 3. Diagnostic Criteria and Treatment Methods

### 3.1. General Data

420 DTC patients admitted from March 2020 to December 2021 are selected. All patients receive surgical treatment and 131I radionuclide treatment. DTC patients are rolled into a LM group and a non-LM group according to the presence or absence of LM. Inclusion criteria are as follows: (1) Those who undergo thyroidectomy and neck lymph node dissection according to the 7th edition of the treatment guidelines of the American Joint Committee on Cancer Staging for thyroid cancer and are pathologically confirmed for DTC. (2) 131I whole body imaging and pathological diagnosis of LM. Exclusion criteria are as follows: (1) Those with other distant metastases. (2) Those with unclear causes of LM. (3) Those with other malignant tumors. (4) Those who are pregnant or breastfeeding. (5) Those with severe liver and renal insufficiency. (6) Those with unclear pathological diagnosis. (7) Those with incomplete clinical data. (8) Those who have not completed regular follow-up.

### 3.2. Diagnostic Criteria

DTC and LM imaging features are shown in Figure 1. The diagnosis of LM-DTC and other distant metastases are carried out by using thyroid tumor pathology, clinical symptoms, serum indexes, 131I whole body imaging, X-ray, and computed tomography (CT) methods. LM-DTC need to meet at least one of the following criteria. (1) 131I whole body imaging suggests abnormal 131I lesions in the lungs of the patient, or other imaging studies support LM. (2) Positron emission tomography (PET)/CT images suggest that the patient's lungs are positive, and other false-positive diseases such as tuberculosis and inflammation are excluded. (3) 131I whole body imaging and PET are negative, but X-ray imaging, CT imaging, and triglyceride (Tg) examination are abnormal. (4) Pathologically confirm pulmonary nodules.

### 3.3. Treatment Methods

Patients need to abstain from iodine-containing food and stop taking levothyroxine tablets or thyroxine tablets for 2∼3 weeks before receiving 131I treatment. Before treatment, all patients receive auxiliary examinations such as blood routine examination, nine items of thyroid function, liver and kidney function, thyroid iodine uptake rate, neck ultrasound imaging, chest X-ray, chest CT imaging, and thyroid static imaging. In the first treatment, 70∼200 mci of nail ablation is given and 200∼230 mci of LM lesions are given. In the state of fasting for 4 hours, 131I is administered orally, 131I whole body imaging is performed 48 hours later, and thyroid hormone suppression therapy is given; 4 days later, it should repeated with the interval of 3∼12 months.

### 3.4. Judgment Basis for Efficacy

The treatment effect is judged as three categories: cure (CR), progesterone-receptor (PR), and no change (NC).

CR is as follows. 131I whole body scintigraphy or PET/CT imaging shows that the patient's LM foci disappear. The serum thyroglobulin level is less than 1.0 *μ*g/L in the state of thyroid stimulating hormone (TSH) suppression and after stimulation without the interference of thyroglobulin antibody (TGAb). Chest radiographs or CT images do not suggest metastatic disease, and no recurrence is found with at least 12 months of follow-up.

PR is as follows. 131I whole-body imaging or PET/CT imaging or chest X-ray or chest CT imaging indicates that the patient had LM lesions, but the number of metastatic lesions is reduced and there is no new increase, and the radiological concentration lesions are reduced and shrunk. Serum Tg levels are consistently higher than 1.0 *μ*g/L and decrease by at least 25% compared to pretreatment Tg levels.

NC is as follows. 131I whole body imaging or PET/CT image or chest X-ray or chest CT image shows that the patient have no new metastases and the serum Tg level decreases by 0∼25% after treatment.

PD is as follows. 131I whole body imaging or PET/CT image or chest X-ray or chest CT image indicates that the patient has increased and enlarged LM lesions, and the newly added metastases have no 131I uptake function and serum Tg levels after treatment increase.

### 3.5. Observation Indicators

Observation indicators are as follows.

1. Clinical data of patients are collected, including patient age, gender, disease course, underlying primary disease, surgical treatment, cervical and mediastinal LNM, lymph node dissection, pathological type, number of lesions, and size of lesions.
2. It should take pulmonary function test, including patient's vital capacity (VC), forced vital capacity (FVC), forced expiratory volume in 1s (FEV1), and maximum ventilation volume (MVV).
3. It should evaluate the clinical effect of 131I-treated patients and judge the effect of the results as CR, PR, NC, and PD according to the evaluation criteria in the previous section.
4. It should collect peripheral venous blood from patients in fasting state, take the upper serum, and store it at −80°C for future use. The detection operation is performed according to the instructions of the ELISA kit, and the absorbance is detected at a wavelength of 450 nm on a Thermo microplate reader. Finally, the detection and calculation of MMP-13 expression level in serum are carried out.
5. The total RNA is extracted from the peripheral blood of patients, and the extracted RNA is reverse transcribed using the miRNA cDNA first-strand synthesis kit. The expression levels of miR-142 and U6 in patients are detected according to the instructions of the miRNA fluorescence quantitative detection kit. The U6 is undertaken as the internal reference gene to calculate the relative expression level of miR-142.

### 3.6. Statistical Analysis

SPSS 19.0 is employed to process and analyse patient data and experimental data. Enumeration data are expressed as (*n* (%)), and chi-square test is for statistical analysis. Measurement data are expressed in the form of (mean ± sd), and statistical analysis is performed using independent samples *t* test. Logistic regression analysis is adopted to analyse the risk factors of LM-DTC patients. Receiver operating characteristic (ROC) curves are drawn for the clinical efficacy of MMP-13 and miR-142 in diagnosing LM in DTC patients. When *P* < 0.05, the difference is statistically significant.

## 4. Diagnostic Efficacy and Evaluation of Clinical Efficacy

Figure 2 shows the univariate analysis of clinical data of LM-DTC. It is clearly evident from Figure 2 that the gender, age, disease course, tumor diameter, pathological type, number of lesions, underlying medical history, cervical LNMs, mediastinal LNM, thyroid capsule invasion (TCI), and ETI are compared between LM-DTC and non-LM patients, and there is no significant difference in gender, age, tumor diameter, number of lesions, and basic medical history between the patients in the LM group and non-LM group. In the LM group, the disease course is longer than 36 months, the pathological type is follicular carcinoma, the cervical and mediastinal LNM, TCI, and ETI are more than those in the non-LM group (*P* < 0.05).

Figure 3 shows the detection of MMP-13 and miR-142 levels in LM-DTC blood. It is clearly evident from Figure 3 that the serum MMP-13 levels in the LM group and non-LM group patients are 135.6 ± 11.3 pg/mL and 75.1 ± 14.0 pg/mL, respectively, and the miR-142 expression levels are 1.14 ± 0.56 and 4.88 ± 0.39, respectively. The serum levels of MMP-13 in the non-LM group are observably lower than those in the LM group, while the expression of miR-142 is much higher (*P* < 0.05).

Table 1 shows the multivariate analysis of LM-DTC. It is clearly evident from Table 1 that the disease course longer than 36 months, the pathological type of follicular carcinoma, cervical LNM, mediastinal LNM, TCI, ETI, and high expressions of MMP-13 and miR-142 are independent risk factors for LM-DTC.

Figure 4 displays the ROC curve of blood MMP-13 and miR-142 in the diagnosis of LM-DTC. It is clearly evident from Figure 4 that the areas under the ROC curves of MMP-13 and miR-142 for the diagnosis of LM-DTC are 0.857 and 0.803, respectively (*P* < 0.05). When the cut-off value of MMP-13 is 143.07 pg/mL, its diagnostic sensitivity and specificity for DTC LM are 95.0% and 89.8%, respectively. When the cut-off value of miR-412 is 1.8, its diagnostic sensitivity and specificity for DTC LM are 85.0% and 82.8%, respectively.

Figure 5 shows the clinical efficacy of 131I in the treatment of DTC without LM and LM. It is clearly evident from Figure 5 that the CR, PR, NC, and PD patients treated with 131I in DTC without LM are 168 (42.0%), 211 (52.7%), 21 (5.3%), and 0 (0.0%), respectively. The CR, PR, NC, and PD patients of DTC LM patients treated with 131I are 6 (30.0%), 10 (50.0%), 3 (15.0%), and 1 (5.0%) patient, respectively. The total cure rates of the LM group and non-LM group are 16 cases (80.0%) and 379 cases (94.8%), respectively, showing no obvious difference in cure rates (*P* > 0.05).

Figure 6 displays the univariate analysis of the clinical effect of 131I in the treatment of DTC. It is clearly evident from Figure 6 that the differences in gender, age, disease course, tumor diameter, pathological type, surgical method, and imaging time are compared between the effective and ineffective patients after treatment. The patients in the IE group are older than 50 years old, the disease course is longer than 36 months, the pathological type is follicular carcinoma, and the patients with LM found at follow-up are more than those in the E group (*P* < 0.05).

Table 2 shows the multivariate analysis of the clinical effect of 131I in the treatment of DTC. It is clearly evident from Table 2 that the age of the patients is older than 55 years, the disease course is longer than 36 months, and the imaging timing are the independent risk factors affecting the effect of 131I in the treatment of DTC.

## 5. Conclusions

This work is to explore the risk factors of LM-DTC and the factors affecting the effect of 131I in the treatment of LM-DTC. The results show that the pathological type of follicular carcinoma, with cervical and mediastinal lymph node metastasis, with a thyroid capsule and external tissue invasion, abnormal expression levels of MMP-13 and miR-142 are risk factors for LM-DTC. MMP-13 and miR-142 can be deemed as auxiliary diagnostic serum biological indicators for DTC or not. However, age, disease course, and imaging timing all affect the therapeutic effect of 131I on LM-DTC patients. Therefore, it is of great significance to focus on DTC patients with the abovementioned characteristics in clinical practice for improving the prognosis of patients.

## Figures and Tables

**Figure 1:** DTC and LM imaging features: (a) 131I whole body imaging; (b) CT imaging; (c) whole body PET/CT imaging.

**Figure 2:** Univariate analysis of clinical data of LM-DTC: (a) difference in gender, age, tumor diameter, number of lesions, etc; (b) difference in thyroiditis, cervical lymph node metastasis, etc.

**Figure 3:** Detection of MMP-13 and miR-142 levels in LM-DTC blood: (a) the level of MMP-13; (b) the expression of miR-142.

**Figure 4:** ROC curve of blood MMP-13 and miR-142 in the diagnosis of LM-DTC: (a) ROC curves of MMP-13; (b) miR-142 in the diagnosis of LM-DTC.

**Figure 5:** Clinical efficacy of 131I in the treatment of DTC without LM.

**Figure 6:** Univariate analysis of the clinical effect of 131I in the treatment of DTC.

**Table 1:** Multivariate analysis of LM-DTC.

Variable	B	SE	Wald *χ*^2^	OR	*95% CI*		*P*
					Lower	Upper	
Constant	1.204	2.056	0.384	3.707	—	—	0.001
Disease course	0.737	0.219	7.813	2.330	0.882	5.017	0.001
Pathological type	2.015	0.108	3.241	7.116	3.517	17.039	0.001
Cervical LNM	1.635	0.843	3.519	7.934	4.036	10.290	0.001
Mediastinal LNM	1.092	0.427	4.517	2.988	1.530	6.718	0.001
TCI	1.356	0.505	10.043	6.452	2.051	12.086	0.001
ETI	1.148	0.384	3.160	2.891	1.369	5.633	0.001
MMP-13	1.567	2.513	0.871	4.990	1.532	7.978	0.001
miR-142	1.343	1.897	1.035	4.614	2.041	6.037	0.001

**Table 2:** Multivariate analysis of the clinical effect of 131I in the treatment of DTC.

Variable	B	SE	Wald *χ*^2^	OR	*95% CI*		*P*
					Lower	Upper	
Constant	2.088	0.336	0.212	9.819	—	—	0.001
Age	−2.039	0.418	2.345	0.202	0.045	0.673	0.005
Disease course	1.947	1.041	0.709	1.343	0.670	2.411	0.001
Pathological type	1.284	0.970	1.457	0.815	0.049	0.557	0.053
Imaging timing	−3.126	0.599	1.668	0.120	0.031	0.352	0.002

## Data Availability

The simulation experiment data used to support the findings of this study are available from the corresponding author upon request.
